The article "Transcranial Electrical Motor Evoked Potential in Predicting Positive Functional Outcome of Patients after Decompressive Spine Surgery: Review on Challenges and Recommendations towards Objective Interpretation" was retracted in 2023. Reasons: signs of a paper mill; suspected computer-generated content; unreliable results or conclusions; lack of ethics approval or compliance.

# Transcranial Electrical Motor Evoked Potential in Predicting Positive Functional Outcome of Patients after Decompressive Spine Surgery: Review on Challenges and Recommendations towards Objective Interpretation

**DOI:** 10.1155/2021/2684855

**Published:** 2021-11-03

**Authors:** Mohd Redzuan Jamaludin, Khin Wee Lai, Joon Huang Chuah, Muhammad Afiq Zaki, Yan Chai Hum, Yee Kai Tee, Maheza Irna Mohd Salim, Lim Beng Saw

**Affiliations:** ^1^Department of Biomedical Engineering, Faculty of Engineering, Universiti Malaya, 50603 Kuala Lumpur, Malaysia; ^2^Department of Electrical Engineering, Faculty of Engineering, Universiti Malaya, 50603 Kuala Lumpur, Malaysia; ^3^Center of Environmental Health and Safety, Faculty of Health Sciences, Universiti Teknologi Mara Selangor, Puncak Alam Campus, 42300 Bandar Puncak Alam, Selangor Darul Ehsan, Malaysia; ^4^Centre for Healthcare Science & Technology, Department of Mechatronics and Biomedical Engineering, Lee Kong Chian Faculty of Engineering and Science, Universiti Tunku Abdul Rahman, Malaysia; ^5^Bioinspired Device and Tissue Engineering Research Group, School of Biomedical Engineering and Health Sciences, Faculty of Engineering, Universiti Teknologi Malaysia, 81300 Skudai, Johor, Malaysia; ^6^Department of Orthopaedic Surgery, Sunway Medical Centre, Malaysia

## Abstract

Spine surgeries impose risk to the spine's surrounding anatomical and physiological structures especially the spinal cord and the nerve roots. Intraoperative neuromonitoring (IONM) is a technology developed to monitor the integrity of the spinal cord and the nerve roots via the surgery. Transcranial motor evoked potential (TcMEP) (one of the IONM modalities) is adopted to monitor the integrity of the motor pathway of the spinal cord and the motor nerve roots. Recent research suggested that the IONM is conducive as a prognostic tool towards the patient's functional outcome. This paper summarizes the researches of IONM being adopted as a prognostic tool. In addition, this paper highlights the problems associated with the signal parameters as the improvement criteria in the previous researches. Lastly, we review the challenges of TcMEP to achieve a prognostic tool focusing on the factors that could interfere with the generation of a stable TcMEP response. The final section will discuss recommendations for IONM technology to achieve an objective prognostic tool.

## 1. Introduction

Spine surgeries (such as posterior spinal instrumentation and fusion, discectomy, and laminectomy) are usually conducted along the spine vertebra that is surrounded by the spinal cord, the nerve roots, and other relevant vascular supply to these elements; thus, spine surgeries pose high risk to the patient concerning the motor and sensory functions [1, 2]. Intraoperative neuromonitoring (IONM) refers to a technology to provide information on the dorsal column somatosensory and corticospinal motor pathway integrity during the surgery [1, 3]. IONM consists of several tests (such as motor evoked potential (MEP), somatosensory evoked potential (SSEP), and other descending neurogenic evoked potentials) which can be utilized to monitor neurologic activities. Benefited from these modalities, surgeons can be notified in a timely manner allowing the possibility or reversing neurologic deficits before these deficits further deteriorate [2–5].

The article "Transcranial Electrical Motor Evoked Potential in Predicting Positive Functional Outcome of Patients after Decompressive Spine Surgery: Review on Challenges and Recommendations towards Objective Interpretation" was retracted in 2023. Reasons: signs of a paper mill; suspected computer-generated content; unreliable results or conclusions; lack of ethics approval or compliance.

Ideally, IONM is applied on a patient that has no neurologic impairment to acquire a meaningful baseline so that any signal deterioration induced by surgical intervention during the surgery could be detected and reversed [6]. IONM is possible to be applied on patients who have neurological deficit preoperatively (due to structural compression to the spinal cord or nerve roots) despite reduced or no response to the IONM. However, when a decompression is performed, the conductivity of the neural structure can be indicated by an improved IONM response; this response holds potential to be valuable information for the surgeon [6]. This paper focuses on reviewing the findings that indicate the prognostic value of improved MEP signals after surgical interventions were conducted.

### 1.1. Brief Introduction to Motor Evoked Potential (MEP)

Motor evoked potential (MEP) functions to monitor the motor function of a patient [7]. Spinal and brainstem motor neurons together with the corresponding peripheral axons constitute a system known as Lower Motor Neurons (LMNs) [8]. The MEP, generated by the firing of LMNs, excites muscle response. To produce the firing of LMNs through external stimulation, pulse train stimulation is utilized to evoke a series of *D*-waves and *I*-waves; a sequential excitatory postsynaptic potential (EPSP) is thus produced. The accumulation of EPSPs, if the firing threshold is achieved, induces the firing of LMNs which in turn results in muscle contraction permitting the acquisition of muscle's MEP. In summary, electrical stimulation from the motor cortex of the brain and muscles will respond to the stimulation by contraction thus producing recordable MEP signals [7, 9, 10].

## 2. The Significance of MEP Improvement

The main purpose of intraoperative monitoring is to prevent nonreversible damage to the neural structure of a patient during surgery. Usually, the most ideal situation to apply IONM is to apply it on patients without neurologic impairment in order to acquire ideal MEP's baseline; thus, any surgical intervention that induces signal deterioration during the surgery can be compared to this baseline and interpreted efficiently [6]. However, MEP can also be applied to patients with neurological deficit preoperatively due to structural compression to the spinal cord or nerve roots, but these could lead to reduced or no response at all to the MEP. Thus, when a decompression is performed, the conductivity of the neural structure could be indicated by an improved MEP response and hence it is conducive to the surgeon [6].

The article "Transcranial Electrical Motor Evoked Potential in Predicting Positive Functional Outcome of Patients after Decompressive Spine Surgery: Review on Challenges and Recommendations towards Objective Interpretation" was retracted in 2023. Reasons: signs of a paper mill; suspected computer-generated content; unreliable results or conclusions; lack of ethics approval or compliance.

The comparison between TcMEP outcomes and pain visual analogue scale (VAS) was shown by Voulgaris et al. [11] on 25 patients' data that have undergone lumbar spinal stenosis surgery for decompressive laminectomy. The patients were evaluated preoperatively with the VAS scale and again postoperatively at a third month and 12th month interval. The IONM modalities adopted were the TcMEP and EMG monitoring. The corkscrew electrodes for MEP were placed at C1–C2 with multipulse current stimulation ranging from 0 mA to 200 mA. Each of the stimulus duration was set from 0.2 ms to 0.5 ms. The muscles' electrodes for MEP and EMG were put according to the level of operations. The MEP improvement criteria were set to exceed 50% of amplitude increment. The Wilcoxon signed-rank test was used as the statistical analysis to compare the presurgery and postsurgery VAS score. Result shows that the mean VAS score demonstrated improvement at the third month follow-up and further improved at the 12th month follow-up as compared to the preoperative score. No patient experienced transient or permanent motor deficit after the surgeries. Among the 25 patients, 17 patients had more than 50% improvement to the MEP response postdecompression and 6 patients exhibited slightly increased response or no changed response, while the remaining 2 were not accommodated with IONM during their surgeries because of the application of an inhalational agent by the anaesthetists. The patients with more than 50% MEP response improvement showed a better VAS score at the 12th month follow-up as compared to the remaining patients.

Visser et al. [6] presented a study of 8 patients out of 74 patients with spinal canal stenosis (*n* = 2), extradural meningioma (*n* = 3), or a herniated nucleus polposus (*n* = 2) that showed significant improvement on MEP responses after decompression of the spinal cord or cauda equina. Out of the 74 patients, 44 patients experienced the onset of neurological symptoms for more than 6 months before the surgery date and 30 patients experienced neurological symptoms for less than 6 months before the surgery date. The stimulus parameter adopted were transcranial voltage stimulation using either Cz–Fz montage with a monophasic pulse train or C3–C4 montage with a biphasic pulse train. Muscle groups without responses remained under monitoring to detect improvement on MEP response after the surgical decompression. Three of the 4 lower limb muscles (quadriceps (L2–L4), tibialis anterior (L4–L5), hamstrings (L5–S1), and gastrocnemius (S1–S2)) were selected depending on the thoracolumbar surgical levels. As a control, the abductor digiti minimi or abductor pollicis brevis was selected. For cervical procedures, the trapezius (C2–C4), the biceps (C5–C6), the triceps (C7–C8), and the extensor of the forearm (C6–C7) or the abductor digiti minimi (C6–C8) were adopted for monitoring. The control for cervical procedures was selected from either the trapezius muscle or orbicularis oris muscle. There was no SSEP modality applied on all the patients. Anaesthetic-wise, a short-acting muscle relaxant was used during intubation together with propofol (4–8 mg·kg^−1^·h^−1^), ketamine (2.5 *μ*g·kg^−1^·min^−1^), and remifentanil (0.05–0.5 *μ*g·kg^−1^·min^−1^). MEP responses were recorded at the start and at the end of the procedures. If the baseline MEP amplitude exceeds 10 *μ*V, the changes of MEP amplitude were computed in percentage. If the baseline MEP amplitude is less than 10 *μ*V or no response at all, the increment of the MEP amplitude (if any) was stated as “response appearance after absence.” A significant improvement to the MEP signal was defined as exceeding 200% increment of amplitude to factor out other factors that affected the MEP amplitudes. Patients' age, gender, medical history, onset of neurologic symptoms, neurologic function before surgery, neurologic function 3 months after surgery, pathology, type of surgery, anaesthetic details during the surgeries, and postoperative blood loss were recorded and analyzed. The muscle motor function (muscle strength, sensory function, neurogenic pain, and walking distance) was analyzed based on the Medical Research Council with a scale from 0 to 5. Any sign of relief from the stated symptoms was defined as neurologic improvement. Out of the 44 patients with more than 6 months of neurologic symptoms, 24 of them showed no improvement of symptoms 3 months after the surgery despite having more than 100% of MEP amplitude increment. Meanwhile, 20 patients from the same group had improvement of symptoms 3 months after the surgery, but none of them had an increment of MEP amplitude for more than 100%. The other 30 patients had neurological symptoms for less than 6 months, and 13 of them had no improvements of symptoms 3 months after surgery and no improvement on MEP amplitude, while 17 of them had improvement of symptoms 3 months after surgery and 6 of them had more than 100% improvement on MEP amplitude. Even though the 8 patients had improvement of MEP amplitude postdecompression, 2 of them had no improvement to their neurological symptoms. A relation (by Visser et al. [6]) was found between the duration of the neurological deficit onset prior to the surgery date; these 2 patients had more than 6 months of neurological deficit as compared to the other 6 patients who had MEP improvement and symptom improvement with only less than 6 months of neurological deficit.

The article "Transcranial Electrical Motor Evoked Potential in Predicting Positive Functional Outcome of Patients after Decompressive Spine Surgery: Review on Challenges and Recommendations towards Objective Interpretation" was retracted in 2023. Reasons: signs of a paper mill; suspected computer-generated content; unreliable results or conclusions; lack of ethics approval or compliance.

Another study by Raynor et al. [12] of 12375 spinal surgeries over 25 years presented the efficacy of multimodality IOM in relation to the outcome of the surgeries. Out of the 12375 patients, IOM signals were spotted to have changes whether the changes were improvements or degradations in 386 patients. The multimodality IOM included descending neurogenic evoked potentials (DNEP), transcranial electrical motor evoked potentials (TcMEP), spontaneous electromyography (EMG), triggered electromyography (TrigEMG), and dermatomal SSEP (dSSEP). The anaesthetic protocol was applied according to the conditions of surgeries, patients, and anaesthetic guidelines, although certain anaesthetic criteria were followed to ensure that the IOM could be performed effectively: halogenated agents were applied not more than 0.5 MAC, NO_2_ usage should be applied less than 50% of the end tidal volume, and no muscle relaxant was used when TcMEP was utilized. The TcMEP used C3–C4 motor cortex scalp electrode montage. The TcMEP was mostly used on upper extremity surgeries and only some on lumbar cases requested by the surgeons. The result showed that of all the changes from the 386 patients with 406 IOM signals' significant events or true positive events, 360 patients' events indicated signal improvement after surgical interventions were conducted. One patient from the 360 improved IOM signals had permanent neurological deficit. The balance 46 events had no improvement to the IOM signals despite the fact that surgical interventions were applied, and out of these instances, 14 patients were confirmed with permanent neurological deficits. The comparison between one patient with the improved IOM signal but permanent neurological deficit and 14 patients that had no signal improvement with true permanent neurological deficit was still statistically significant. However, this study did not specify the improvement criteria and which modalities exactly were indicated to have IOM signal improvement by the authors.

Wang et al. [13] presented a finding from degenerative cervical compressive myelopathy (CCM) cases from 59 patients that went through laminoplasty or laminectomy procedures with reliable MEP baseline from December 2013 until April 2015. Patients with no reliable or no MEP readings at all were secluded from the study. The selected 59 patient's data were categorized into a group with more than 50% of MEP improvement, a group with less than 50% MEP improvement or considered not significant, and a group with MEP degradation. Patients were assessed preoperatively with the mJOA scale and postoperative evaluation of motor, sensory, and pain a week after and 6 months after surgery with the mJOA scale. Both MEP and SSEP modalities were used for monitoring. Information regarding the MEP settings adopted for monitoring, and the muscles used to monitor the MEP responses, was absent from the research. The MEP responses were recorded predecompression, postdecompression, and throughout the surgery. The anaesthesia protocol adopted was TIVA without muscle relaxant or inhalation agents with the use of propofol (5–8 mg·kg^−1^·h^−1^), remifentanil (0.05–2 *μ*g·kg^−1^ min^−1^), and fentanyl (5–6 *μ*g·kg^−1^). One-way ANOVA using SPSS 19.0 (SPSS, Inc., Chicago, IL, USA) software was used for statistical comparison analysis with *p* < 0.05 as the statistical difference. The results showed that 21 patients had MEP improvement postdecompression with a mean MEP improvement rate at 140 ± 76%, 32 patients had no significant MEP changes, and six patients had deteriorated MEP signals. The mJOA improvement rate was significantly better for patients that had MEP improvement compared to the group that had no significant changes to the MEP response (59.5 ± 4.2% vs. 48.9 ± 3.9%, *p* < 0.05) and the improved MEP group against the deteriorated MEP response group (59.5 ± 4.2% vs. 40.6 ± 7.4%, *p* < 0.05). The authors also highlighted that MEP amplitude was more effective compared to the MEP latency or SSEP modality in predicting the outcome of the surgery.

The article "Transcranial Electrical Motor Evoked Potential in Predicting Positive Functional Outcome of Patients after Decompressive Spine Surgery: Review on Challenges and Recommendations towards Objective Interpretation" was retracted in 2023. Reasons: signs of a paper mill; suspected computer-generated content; unreliable results or conclusions; lack of ethics approval or compliance.

Another study was made by Wi et al. [14] on 29 improved IONM of spine cases compared to the baselines out of 317 cases with IONM of spine cases and their clinical significance. The surgeries' IONM data were chosen between January 2013 and May 2017. The modalities that were used as monitoring tools were MEP and SSEP. The spine cases of the 29 patients included cervical myelopathy (22 patients), neurofibroma C1 (1 patient), thoracic myelopathy (5 patients), and neurogenic tumour L5–S1 (1 patient). The MEP monitoring was performed bilaterally from the deltoid, triceps, and thenar muscles for the upper extremities, while for the lower extremities, the tibialis anterior and abductor hallucis were used. Meanwhile, the SSEP was stimulated from the median nerve for upper limbs and posterior tibial nerves for the lower limbs. No specific MEP stimulation parameters were mentioned, and only the stimulation was given accordingly for each patient to obtain acceptable responses. The IONM events were recorded at the beginning of the surgeries as the baseline, before change, during change, after change, and throughout the main procedure. The anaesthesia protocol utilized the TIVA protocol with propofol (4.5 *μ*g/mL) and/or remifentanil (1.7 ng/mL) with the usage of a short-acting muscle relaxant during intubation. Patients' data for analysis were selected preoperatively and 3 months postoperatively. The data included the measurement of Motor Index Scoring System (MISS), the Short-Form 36 Health Survey Questionnaire (SF-36), the Japanese Orthopaedic Association (JOA) Cervical Myelopathy Evaluation Questionnaire (JOACMEQ), and Neck Disability Index (NDI) for cervical myelopathy patients, the JOA for thoracic myelopathy patients, and the JOA Back Pain Evaluation Questionnaire and Oswestry Disability Index for lumbar disorder patients. The statistical analysis was performed by using IBM SPSS software version 23.0 (IBM Corp., Armonk, NY, USA) by comparing the preoperation and postoperation by using the Wilcoxon rank-sum test while the improvement rate of MISS and SF-36 was compared by using the Kruskal-Wallis test given the threshold for significance at *p* < 0.05. It was found that 29 patients exhibited improvement to the IONM signals from the recorded data. Two patients with early death (which was unrelated to the surgery) were excluded from the analysis. Ten patients had MEP-only improvement with 8 of them exceeding 100% increment in amplitude, one of them having a response appearance, and one of them having both 100% amplitude increment and response appearance. Twelve patients had SSEP-only improvement with 10 of them having an increase more than 100% increase in amplitude, one of them having more than 6% of decrement of latency, and one of them having both 100% of amplitude increment and 6% of latency decrement. Five patients had both MEP and SSEP improvement. It was found that the MISS improvement rate was significantly better in the group that had MEP improvement only compared to the other two groups while the SF-36 improvement rate was significantly better in the group that had SSEP improvement only compared to the other two groups. It was concluded by the authors that the improvement of IONM signals was conclusive to show that the decompression of the spinal cord is successful and can be valuable information to the surgeon. However, several limitations were mentioned; for example, the study did not compare the group which had no IONM improvement and the group with IONM improvement and the sample size was relatively small and included one lumbar case.

The article "Transcranial Electrical Motor Evoked Potential in Predicting Positive Functional Outcome of Patients after Decompressive Spine Surgery: Review on Challenges and Recommendations towards Objective Interpretation" was retracted in 2023. Reasons: signs of a paper mill; suspected computer-generated content; unreliable results or conclusions; lack of ethics approval or compliance.

Barley et al. [15] reported a case of a 15-month-old boy with a tethered spinal cord extending through the entire cord and a worsening scoliosis. The patient had greater motor weakness on the left upper extremities than on the right upper extremities and weak lower extremities. The tethered cord release and spine correction procedures were performed with the assistance of NIOM. The baseline of TcMEP and SSEP of posterior tibial nerves and ulnar nerves was obtained. TcMEP was stimulated on C1 and C2, and monitoring was performed bilaterally on the quadriceps femoris, tibialis anterior, gastrocnemius, sphincter, abductor pollicis brevis (APB), and abductor hallucis. The stimulation for TcMEP was set from 145 mA to 187 mA for the left extremities and from 175 mA to 200 mA for the right extremities. The only TcMEP response obtained during baseline was on the right-side APB, and the SSEP showed no response during baseline acquisition. It was found that the TcMEP signal on the left APB appeared immediately with increased amplitude after the completion of the cord untethering. Furthermore, the right-side APB also had increment in amplitude, but no SSEP changes were obtained after the detethering procedure. Afterwards, the patient exhibited observable left upper extremity improvement notified by the family and the physicians which supported the outcome of the TcMEP response obtained after the cord detethering procedure.

The next study that researched on the usefulness of the MEP response as a prognostic tool for spine surgeries was conducted by Dhall et al. [16]. The 32 patients' data that were selected had decompression and instrumented stabilization surgeries. The IONM modalities that were used for the surgeries were EMG, TcMEP, and SSEP. The TcMEP stimulation parameters used were double train with a total of 9 pulses, 50 ms pulse width, 1.7 ms interstimulus, 13.1 ms ISI, and constant voltage with intensity that ranged from 100 V to 1000 V. The authors used anodal stimulation that stimulates C1 to acquire responses on the right side and C2 to obtain responses on the left side. For the anaesthetic protocol, the centre where the data were collected used propofol 120 mcg/kg/min, fentanyl 100 mcg/h, and 1.0% or 0.5 MAC sevoflurane with the aim of obtaining more than 85 mmHg of mean arterial pressure (MAP). The baselines were obtained before the patients were positioned and after the patients were positioned prior to surgeries. The end results of the MEP responses were compared with the axial Magnetic Resonance Imaging (MRI) grade of the Brain and Spinal Injury Centre (BASIC) score. The BASIC score basically ranged from grade 0 that indicates no injury to the spinal cord to grade 4 with more severe spine injury. The American Spinal Injury Association Impairment Scale (AIS) grading was performed before and after surgeries upon discharge, and this was compared with the MEP outcome with the Mann-Whitney *U* test. It was found that the presence of MEP was highly correlated with the AIS at discharge that showed that the patients with present MEP had a higher AIS grade as compared to the patients with absent MEP. The correlation of MEP and BASIC scores was implemented by using the Spearman correlation, and it was found that patients that had absent MEP had higher BASIC scores significantly compared to the patients that had present MEP.

The article "Transcranial Electrical Motor Evoked Potential in Predicting Positive Functional Outcome of Patients after Decompressive Spine Surgery: Review on Challenges and Recommendations towards Objective Interpretation" was retracted in 2023. Reasons: signs of a paper mill; suspected computer-generated content; unreliable results or conclusions; lack of ethics approval or compliance.

Piasecki et al. [17] did a prospective study of the predictive value of the MEP outcome of patients that had lumbar spinal stenosis decompression surgeries. As much as 24 consecutive patients' data were used for the study, which were collected within a 28-month period, and all of them had central spinal stenosis without lateral recess stenosis. But only 18 patients' data were selected since they were the only patients that had complete follow-up records. The adopted IONM modalities were TcMEP and lower limb SSEP. The SSEP data were not adopted for the study as the stimulation of the posterior tibial nerve only concerned one nerve root which was the S1 nerve root. The TcMEP stimulation used 50 V to 150 V intensity, biphasic stimulation, 500 Hz of 5 to 7 train pulses, and 1 ms intertrain. The TcMEP corkscrew electrodes were placed at C1–C2. The anaesthetic protocol adopted mainly TIVA with sufentanil and propofol, while a muscle relaxant was only used during intubation. The patients were assessed by using the Zurich Claudication Questionnaire (ZCQ) which was a self-assessment score before surgery (baseline) and after surgery (at 8 months after surgery and 29 months after surgery). The ZCQ scores were obtained by dividing the relative change scores (obtained by patients answering self-assessment questionnaire after surgery) with the baseline scores, and if the score was more than 0.5, it indicated significance for the study. The ZCQ scores were used to be compared with the outcome of the MEPs. The muscles used were dependent upon the level of the surgeries with the bilateral tibialis anterior and abductor hallucis as considerations. One upper limb muscle was used as the reference. The area under the curve of the MEP was used as the measurement tool to compare between the baseline value and after the full decompression value. It was mentioned that 20% of improvement was significant. The outcome of the MEP values showed that eight patients had improvement of more than 20%, three patients had MEP improvement of less than 20%, and 7 patients showed no MEP improvement. Fisher's exact test and the linear Pearson correlation were the statistical analysis tools used accordingly. It was found that by dichotomizing the data, the MEP improvement correlates with the ZCQ score at the early follow-up, while there was only a minor correlation between the 2 at the latest follow-up.

The article "Transcranial Electrical Motor Evoked Potential in Predicting Positive Functional Outcome of Patients after Decompressive Spine Surgery: Review on Challenges and Recommendations towards Objective Interpretation" was retracted in 2023. Reasons: signs of a paper mill; suspected computer-generated content; unreliable results or conclusions; lack of ethics approval or compliance.

He et al. [18] presented a case report of a 60-year-old male patient that had a percutaneous endoscopic lumbar discectomy with the aid of IONM of MEP and free-running EMG modalities. The patient had more than 10 years of low back pain symptom with progressive left lower limb radicular pain and numbness a week before the procedure was done. The muscle strength evaluation of the quadriceps and first toe was 4/5 grades. The diagnosis of the patient imaging showed that the lumbar L2/L3 nerve roots on the left had been compressed by the herniated disc. The IONM recording electrodes were placed at the iliopsoas, rectus femoris, tibialis anterior, and medial gastrocnemius muscles bilaterally. There were no fluctuations of free-running EMG signals during the procedure. However, the MEP amplitude was increased after decompression was done. The patient presented a relieved pain of the low back and leg immediately after he was awake. This case report showed that the MEP could provide immediate feedback on the nerve root decompression effectiveness.

Another case report was presented by Rodrigues et al. [19] of a 22-year-old male athlete who had a decompression surgery after having lumbar pain symptom over 6 months. The patient was examined for muscle strength and showed grade 4/5 of the dorsiflexion of the right foot and hypoesthesia in L5 and S1. The surgery was done with the help of IONM of lower limb SSEP, TcMEP, free-running EMG, and stimulated EMG. The lower limb SSEP monitoring was done by stimulating the bilateral tibial nerve and recorded on the Cz–Fz on the scalp, while the stimulation for the MEP was done on the C3–C4 on the scalp and the recording was done on L3, L4, L5, S1, and S2 myotomes. The anaesthetic protocol utilized was the TIVA protocol with propofol and remifentanil. It was then found that an increment of MEP response amplitude was as much as 30% from the baseline value right after the discectomy procedure. The patient was able to return to a competitive level after a month of surgery.

Table 1 summarizes the findings of studies that proved IONM signal improvement which is correlated with the patients' positive outcome after surgery. If IONM signal improvement can be used as a guidance to indicate actual improvement, it will be valuable to the surgeons during the surgery to determine the depth of decompression which could help to reduce the surgery time and hence lower the risk of nerve injury.

The article "Transcranial Electrical Motor Evoked Potential in Predicting Positive Functional Outcome of Patients after Decompressive Spine Surgery: Review on Challenges and Recommendations towards Objective Interpretation" was retracted in 2023. Reasons: signs of a paper mill; suspected computer-generated content; unreliable results or conclusions; lack of ethics approval or compliance.

It is difficult to measure the exact success rate for TcMEP as a prognosis tool because different studies used different improvement thresholds to show significant improvement. Some papers presented that the TcMEP amplitude after the decompression needs to be more than 50% than the baseline reading to imply actual clinical improvement [11]. Another study showed that the TcMEP amplitude needs to have more than 200% for improvement to happen to overcome the influence of anaesthesia that is used during intubation which could dampen the baseline TcMEP response and hence mislead the surgical team into thinking that there is improvement even though there is not any [6]. Improvement of more than 20% on the area under the curve (AUC) of the TcMEP signal is another indicator used by Piasecki et al. [17], while other studies only mentioned that the improvement of the TcMEP signal is correlated with the postsurgery clinical outcome without mentioning the parameters and the improvement criteria that they used [12, 13, 15, 16, 18, 19].

There are several research questions that can be derived from the previous paragraph. Since there are either 50% or 200% amplitude improvement criteria or 20% of AUC increment, it shows that there are no single universal criteria established that can be used to inform the surgeons that improvement has been achieved intraoperatively. This phenomenon was also presented by [20] that the rate of trial-to-trial variability of MEP is high from one response to another. Visser et al. [6] mentioned that the establishment of a good baseline reading is crucial and yet difficult to generate because of anaesthetic factors with the use of a short-acting muscle relaxant during intubation. The initial responses could be perceived as baseline reading even though it is still under anaesthetic influence and hence could cloud the judgement of whether the final TcMEP response obtained has improved or not.

In the next section, we will review the factors that could influence MEP response so that we could make a suggestion on the utilization of MEP response as a prognostic tool intraoperatively.

### 2.1. Factors Influencing MEP Response

MEP is influenced by various factors, and it is important to identify these factors because if these factors are believed to be affecting the reliability of MEP response readings, the study of the MEP response improvement might not produce accurate favourable results. The factors influencing MEP are generally anaesthesia, the stimulation parameters used by the IONM personnel, electrode placements, surgical interventions, anatomy, physiology, and the technical specialist handling the IONM machine.

The article "Transcranial Electrical Motor Evoked Potential in Predicting Positive Functional Outcome of Patients after Decompressive Spine Surgery: Review on Challenges and Recommendations towards Objective Interpretation" was retracted in 2023. Reasons: signs of a paper mill; suspected computer-generated content; unreliable results or conclusions; lack of ethics approval or compliance.

#### 2.1.1. Anaesthesia

Since the MEP signal is generated by the contraction of muscles when the motor cortex is stimulated, the usage of neuromuscular blockade or muscle relaxant which blocks the transmission of the neurotransmitter causing the patients' reflex movements to be paralyzed should be avoided [8, 21].

Although inhalational anaesthetic agents such as desflurane and isoflurane have advantages such as rapid induction for sedation and recovery with low solubility, Malcharek et al. [22], Lo et al. [23], Pechstein et al. [24], and Tamkus et al. [25] had presented that the failing effects towards MEP response were correlated with the use of inhalational anaesthetic agents. Malcharek et al. [22] found out in their study to compare the effect of anaesthesia particularly between the combination of propofol/remifentanil and the combination of desflurane/remifentanil that the desflurane had a dampening effect on the amplitude of the MEP responses.

On the other hand, Lo et al. [23] reported that the MEP was plausible to be obtained within a suitable desflurane “concentration window” which was 0.5 maximum alveolar concentration (MAC) with 60% of NO_2_ even though there was one patient that had nonreadable MEP response. Pechstein et al. [24] had only one successful MEP signal outcome when isoflurane and NO_2_ were used together with alfentanil compared to the group that had the TIVA protocol with the combination of propofol and alfentanil with the outcome of 15 out 17 successful MEP signals. When they applied only the NO_2_ to the TIVA group 10 minutes before all the tests were completed, they found that the MEP amplitudes were dropped to more than 40% compared to the baseline.

A study conducted by Tamkus et al. [25] involved a large number of samples which were 1814 patients mixed with patients that had preoperative motor deficits and patients with no preoperative motor deficits. They studied the false positive rates for MEP recordings by using inhalational agents and TIVA. False positive was defined as the MEP recording which is observed to be abnormal but not associated with intraoperative or postoperative motor deficits [25]. It turned out that the false positive rates were higher in the inhalational agent group compared to the TIVA group.

Meanwhile, Ubags et al. [26] conducted a study on different concentrations of propofol usage and the effects on the MEP responses had showed that the higher the dosage of propofol used, the more dampening it will impose on the MEP responses as compared to the effect of using NO_2_. Furthermore, a study by Kawaguchi et al. [27] also supported the claim that MEP response excitability is dependent upon propofol dosage in which they showed that MEP response latency had not been significantly influenced by the propofol concentration, but the MEP response amplitude was increasing with the decrement of the propofol infusion rate.

The article "Transcranial Electrical Motor Evoked Potential in Predicting Positive Functional Outcome of Patients after Decompressive Spine Surgery: Review on Challenges and Recommendations towards Objective Interpretation" was retracted in 2023. Reasons: signs of a paper mill; suspected computer-generated content; unreliable results or conclusions; lack of ethics approval or compliance.

Total intravenous anaesthesia (TIVA) using propofol is the common anaesthesia protocol for a successful MEP monitoring [22]. Even though inhalational agents are possible to be used for MEP monitoring, the TIVA protocol is still advisable to be used because various studies have shown that inhalational agents cause a more suppressive effect on the MEP responses compared to the TIVA protocol [22, 24, 25, 28, 29]. Higher concentrations of propofol were shown to suppress the MEP responses, but it goes with the rule that the deeper the anaesthesia is, the lower the MEP responses will be and the lighter the anaesthesia is, the higher the MEP responses will be [8]. With certain stimulus parameter adjustments which will be presented in the following section of this paper, MEP can be obtainable by using propofol even though it was shown that propofol also has some suppressive effects on the MEP responses [24, 26]. A summary of anaesthetic consideration done by Leppanen [30] is shown as follows:

1. NO_2_ ≤ 50%
2. Isoflurane: not to be used or 0.2 to 0.5%
3. Propofol: less than 200 *μ*g/kg/min
4. Fentanyl: continuous infusion
5. Muscle relaxant: not to be used

#### 2.1.2. Stimulation Parameters

There is no standardized protocol for stimulation to obtain MEP [8]. Stimulation parameters include stimulation intensity, number of pulses, pulse duration, single or train stimulation, constant-current or constant-voltage stimulation, anodal or biphasic stimulation, and other stimulation parameters [1, 8, 24, 26, 31–33].

The number of stimulation pulses was shown to have significant contribution to lowering or increasing the stimulus threshold to ignite MEP response [34]. Ubags et al. [26] tested the obtainability of MEP response by using two-pulse MEP stimulation, and the result showed that the MEP responses were obtainable 100% by using two pulses with the propofol-induced protocol. Pechstein et al. [24] applied different numbers of stimulation pulses (1–5 pulses), and it was presented that the amplitude of the MEP responses increased with the increasing number of pulses. However, latencies were not affected significantly by the number of pulses [24].

The article "Transcranial Electrical Motor Evoked Potential in Predicting Positive Functional Outcome of Patients after Decompressive Spine Surgery: Review on Challenges and Recommendations towards Objective Interpretation" was retracted in 2023. Reasons: signs of a paper mill; suspected computer-generated content; unreliable results or conclusions; lack of ethics approval or compliance.

As a summary from combined authors, if more stimulation pulses are used:

1. The latency threshold to obtain the MEP response will be reduced which means that the MEP response will appear sooner on the recording graph [8, 10, 35]
2. The MEP response amplitude will become larger [8]
3. There will be more polyphasic parameters produced on the MEP response signal, thus prolonging the duration of response [8]
4. There will be increased likelihood of achieving the stimulation threshold [1]

Increasing stimulation intensity enhances the current field size and activates the subcortical white matter motor tracts at the bend of the axon exiting the grey matter [8]. This situation is acceptable if the monitored structures are below the foramen magnum such as the spine [1]. If the monitored structures are within the pyramidal tract in the white matter, it is advisable to use minimum MEP stimulus intensity so that any changes within these structures during, for example, brain tumour excision surgeries could be identified [36]. Response duration would also be increasing when stimulation intensity is increased [35].

Shigematsu et al. [32] introduced a method to increase the MEP response recording by using tetanic stimulation at single and multiple peripheral nerve sites. The tetanic stimulation at the posterior tibial nerve, for example, shown in the study a second before the MEP stimulation was evoked enhanced the MEP response at the abductor hallucis muscle which is the muscle innervated from the tibial nerve. It was mentioned by Shigematsu et al. [32] that this technique is suitable for patients with preoperative neurological deficit and patients with neuromuscular anaesthesia blockade.

#### 2.1.3. Electrode Placements

The specific muscles correspond to specific spinal cord levels for efficient MEP monitoring purposes; for example, if the surgery takes place in the lumbar region, generally electrode placement of the leg muscles takes place at TA and AH [37]. The distance between recording electrodes (between active and reference electrodes) and the positioning of the recording electrodes on the muscle could also influence on the amplitude size and latency of the MEP response [38]. MEP response latency was found to be more delayed when the different electrodes were placed at a more distal location of the muscle. It was also recommended by Chomiak et al. [38] to position the recording MEP electrodes at the motor end plate zone and at the distal myotendinous junction to obtain significant MEP response.

The common scalp electrode montage to elicit MEP is C3–C4, but different montages could also lead to different outcomes to the MEP response [39]. Ryosuke et al. [39] simulated the scalp electrode montage from three different montages which were C3–C4, C1–C2, Cz–inion, and Cz–forehead in order to find out the best montage to elicit lower extremity MEP efficiently. The test was conducted on the 3D model of the head, and with finite element analysis, the tests were conducted. It was found that the Cz–inion scalp electrode montage produced MEP for lower extremities with a lower stimulus threshold. These findings are correlated with the homunculus representation of the cortex.

The article "Transcranial Electrical Motor Evoked Potential in Predicting Positive Functional Outcome of Patients after Decompressive Spine Surgery: Review on Challenges and Recommendations towards Objective Interpretation" was retracted in 2023. Reasons: signs of a paper mill; suspected computer-generated content; unreliable results or conclusions; lack of ethics approval or compliance.

The homunculus was developed by Penfield et al. [40] through a lengthy experiment of electrical stimulation to the brains of their patients in order to identify or map the location of which part of the muscles or sensations responded to which part of the brain that was stimulated. Catani [41] had simplified the findings by Penfield et al. [40] with representation of the motor stimulations for different body parts with colour coded. The homunculus shows that the primary motor cortex area of the brain that controls the lower limbs is located towards the medial side of the brain, while the control of the upper limbs is located towards the lateral side of the primary motor cortex [42]. The more complex the movement of the muscle is, the larger the area of the motor cortex involved to control it: just to exemplify, the hand consists of a larger motor cortex area than the legs because of the complex movement it can produce.

Insulation such as a fat layer between the stimulating electrodes on the scalp affects the depth of electrical penetration towards the motor cortex thus influencing the recorded MEP response [43]. The use of peg screw electrodes for stimulation on the scalp could reduce the stimulus threshold because the current passes through the scalp more effectively rather than using corkscrew electrodes where the stimulation current spreads laterally because of the high resistivity of the skull [44–46]. However, the peg screw requires microdrilling before its insertion; this drilling has to be conducted with care to prevent the drilling from penetrating the skull even though the risk is minimal [45].

#### 2.1.4. Surgical Interventions, Anatomy, and Physiology

Temperature affects the MEP response: low temperature increases the latency of the response while higher temperature reduces the latency of the response [8]. The source of temperature changes might stem from the patient's body temperature, or specific muscles' or limbs' temperature, or the temperature of the exposed spinal cord during the surgery [8]. Temperature can also affect MEP indirectly by changing the pharmacokinetics and pharmacodynamics of anaesthetic agents where a study showed that decreased temperature can cause increased concentration of propofol and reduce the bispectral (BIS) index value thus reducing the amplitudes of MEP responses [47]. Other effect of temperature on MEP response is that low temperature could obliterate MEP response while increasing the temperature could revive the MEP response [37].

The article "Transcranial Electrical Motor Evoked Potential in Predicting Positive Functional Outcome of Patients after Decompressive Spine Surgery: Review on Challenges and Recommendations towards Objective Interpretation" was retracted in 2023. Reasons: signs of a paper mill; suspected computer-generated content; unreliable results or conclusions; lack of ethics approval or compliance.

In the study conducted by Kanemaru et al. [48] whereby MEP was performed on patients that underwent descending aortic replacement (DAR) and thoracoabdominal aortic replacement (TAAR) surgeries, they showed that when the patients were put through deep hypothermic circulatory arrest (DHCA) (12°C-22°C), the MEP response disappeared. The MEP amplitude was then increased to more than 50% during the rewarming process when the body temperature reached approximately 34°C. Another similar study was made by Shinzawa et al. [49] that the MEP latencies in both the abductor pollicis brevis (APB) and abductor hallucis (AH) muscles which were tested were inversely proportional to the temperature. It was also found that the AH muscles or the leg muscles had a slower rate of MEP amplitudes' increment during the rewarming process compared to the hand muscles or APB muscles. These studies indicated that the body temperature of the patient should be kept close to the normal human body temperature for MEP monitoring to function well.

MEP response is also subjected to surgical manipulations [50]. MacDonald et al. [51] had elaborately presented the surgical interventions that affected the MEP responses during their study which were as follows:

(1) Hypotension:
  - It is defined as the mean arterial pressure that fells below 60 mmHg
  - Any reduction to MEP responses in the study had considered raising the blood pressure. If there were no other interventions involved in the deterioration of MEP responses, raising blood pressure had shown to bring restoration to MEP responses
(2) Ischemia:
  - Leg ischemia was shown in one of the cases in the presented study which was caused by femoral artery pressure to deteriorate the leg MEP responses. Pelvic support was repositioned and MEP responses gradually returned except the protracted right TA's MEP
(3) Spinal cord contusion:
  - Spinal cord contusion due to instrumentation could cause MEP response deficit
  - As shown by MacDonald et al. [51], placement of the hook into one thoracic vertebra in one of the cases caused disappearance of bilateral leg MEP. Removal of the hook afterwards brought back the MEP responses
  - Another case presented with an overcorrection done had bilateral leg MEP disappearance. The rod was released and the MEP response was returned
  - An idiopathic scoliosis case had disappearance of MEP after discectomy during anterior release. The patient was positioned in lateral flexion. After the patient was straightened, the MEP reappeared

Anatomical factors of the patients could also affect the MEP response. One of the most important practices to perform before any surgical interventions are made is to obtain the best MEP response baseline, and failure to obtain this important information can be caused by preoperative motor function or motor power deficit [52]. This means that the lower the motor power is, the less chance it is to obtain a successful reading of MEP response.

The article "Transcranial Electrical Motor Evoked Potential in Predicting Positive Functional Outcome of Patients after Decompressive Spine Surgery: Review on Challenges and Recommendations towards Objective Interpretation" was retracted in 2023. Reasons: signs of a paper mill; suspected computer-generated content; unreliable results or conclusions; lack of ethics approval or compliance.

Age is also a factor that could affect MEP response as studies showed that a paediatric patient at the age below 7 years has a lower successful rate of producing reliable MEP readings due to the electrophysiologic immaturity of the corticospinal tract which is considered fully developed generally at the age of 10 years old [33, 53].

The number of nerve innervations towards the target muscle represents the sensitivity of the MEP readings as shown in various studies [52, 54]. As shown by Kim et al. [52], the AH muscle is reported to achieve a higher successful rate in producing MEP response as the baseline than the AT muscle, while Yue et al. [54] presented that the event of foot drop postoperatively could be determined from the monitoring of the AT muscle rather than the AH muscle. These two events were deducted as there are more nerves that innervate towards the AH muscle, making it less sensitive to motor power deficit or nerve injury than the AT muscle which has a lower number of nerves that innervate towards it [52].

#### 2.1.5. Technical Specialist Handling the IONM Technology

The team that handles IONM during the surgery plays an integral role in providing reliable interpretation of signals to the entire IONM team even though it is not a direct factor that affects the MEP signal characteristics. The IONM team as defined in Kim et al. [55] consists of the surgeon, clinical neurophysiologist, anaesthesiologist, and monitoring technologist.

Kim et al. [55] claimed that the majority of the IONM signals' changes primarily stem from faulty machine, inappropriate IONM machine settings, changes in the anaesthetic regime, and inconsistent hemodynamic state and are not entirely due to neural damage. These factors could be minimized or eliminated by the expert evaluation and analysis of the experienced neurophysiologist resulting in the reduction of false positive and false negative rates.

In order to prevent neural damage, the neurophysiologist or the monitoring technologist has to interpret the changes or the drop of the signal. The variety of alarm criteria to the MEP signal alone within the literature has led the neurophysiologist to identify the best alarm criteria to suit the situation of the surgery. For instance, Weinzierl et al. [50] proposed to use 50% drop of MEP response amplitude if the surgery is considered less risky and less aggressive by the surgical team and 80% drop of MEP response amplitude if the surgery is more complicated. However, the authors highlighted that if 80% drop of MEP response amplitude was used as their alarm criteria in their studies, 2 of the patients that developed postsurgery motor deficit will be missed out.

The article "Transcranial Electrical Motor Evoked Potential in Predicting Positive Functional Outcome of Patients after Decompressive Spine Surgery: Review on Challenges and Recommendations towards Objective Interpretation" was retracted in 2023. Reasons: signs of a paper mill; suspected computer-generated content; unreliable results or conclusions; lack of ethics approval or compliance.

Another example that requires the neurophysiologist or the monitoring technologist to be equipped with new findings and knowledge in the IONM research area is the usability of certain IONM modalities for certain procedures. For example, Pajewski et al. [56] recommended that no MEP and SSEP monitoring should be used in simple lumbar discectomy or decompression as the modalities would slow down the operation time and prevent muscle relaxation. Meanwhile, He et al. [18] presented that the MEP is beneficial in detecting improvement in MEP intraoperatively which correlated with the relief of symptoms postoperatively. The MEP could also be useful in lumbar procedures with the appropriate MEP monitoring on the tibialis anterior and extensor hallucis longus to prevent foot drop [57]. The researches from He et al. [18] and Lieberman et al. [57] seem contradicting to the proposal made by Pajewski et al. [56], but in the end, it is up to the IONM team to decide on how they would approach the surgeries based on these recommendations from the literatures.

#### 2.1.6. Summary for Factors Influencing MEP Response

Most of the factors influencing MEP response presented in Section 2.1 are already well known and standardized. However, IONM personnel (surgeon, anaesthetist, and technician) acceptance and interpretations towards the standardized knowledge on MEP might vary. Communication within the team is the key to maintain the parameters as steady as possible, so that the IONM can be used solely to analyze the condition of the neural integrity. If communication fails, the IONM technician will have to try to adapt with the patient's physiological changes due to, for example, the anaesthesia fluctuations by adjusting the stimulation parameters, and the adjustment requires skills and experience from the technician himself/herself. These show how each factor is interrelated with one another. We summarized that in order for MEP to be used successfully as an indicator of positive outcome postsurgery, these influencing factors should be maintained to keep the nonsurgical factor from interfering with the interpretation of the MEP.

The article "Transcranial Electrical Motor Evoked Potential in Predicting Positive Functional Outcome of Patients after Decompressive Spine Surgery: Review on Challenges and Recommendations towards Objective Interpretation" was retracted in 2023. Reasons: signs of a paper mill; suspected computer-generated content; unreliable results or conclusions; lack of ethics approval or compliance.

## 3. Discussion

In Malaysia, IONM is usually conducted by IONM technicians from companies that distribute medical devices to the hospitals. There are no specialized neurophysiologists behind every IONM technician to give advices and analyze the IONM signals in depth. The IONM technicians in Malaysia do not necessarily have the specific certificate or qualification in IONM. The companies rely on training for product use conducted by their respective IONM technology supplier or manufacturer, and some may go further by attending IONM conferences conducted worldwide. The IONM technicians in Malaysia need to cope with the technology and become the interpreter or intermediary between the IONM technology and the medical practitioners such as the surgeon and the anaesthetist inside the operation theatre during surgery. It is already challenging to alarm the surgeons and at the same time not limit the surgeons conducting their task. At the same time, apart from inspecting whether the patient's spine integrity is still intact, the surgeons desire to know if they can expect any positive functional outcome to their patients during the surgery through IONM.

Figures 1 and 2 show MEP baseline and after decompression, respectively, of a patient that underwent microendoscopic discectomy of L4/L5. The patient complained of back pain and left leg pain, with no motor weakness, and was diagnosed with lumbar disc prolapse at L4/L5. The percentages of signal peak-to-peak amplitude increments are circled in Figure 2. The amplitude increments are shown to be more than 200% in seven channels and 24% in channel LM4. It is difficult to suggest that the patient will incur positive functional outcome from these signals.

Unlike the alarm criteria, the literatures have established alarm criteria that can be used by the neuromonitoring technologist in live surgery even though there are differences between the studies, whether it is 50% MEP signal drop [50] or 80% MEP signal drop [58], or even with all-or-nothing criteria [1], the IONM technicians can choose the criteria based on their interpretations and situations during the surgery. Alarm criteria can be established since the signal drop can only range from 0% to 100% from the baseline reading.

The increment of the MEP signal can be more than 100% as shown in Figure 2. Based on Table 1, if improvement criteria such as 50% [11] are used, all of the channels in Figure 2 will be noted as improved, even though the only focus is on L4/L5 since that is where the disc prolapse and the patient experience pain only on the left leg. Another example based on Table 1, if 200% increment [6] is chosen as the improvement criteria, all channels will be presumed as having improvement except for channel LM4 that only exhibits 24% of increment. In Sunway Medical Centre, we have experienced many IONM events which were similar to what is shown in Figures 1 and 2, which is why the current literatures' recommendations on the improvement criteria cannot be used for all of the cases.

The article "Transcranial Electrical Motor Evoked Potential in Predicting Positive Functional Outcome of Patients after Decompressive Spine Surgery: Review on Challenges and Recommendations towards Objective Interpretation" was retracted in 2023. Reasons: signs of a paper mill; suspected computer-generated content; unreliable results or conclusions; lack of ethics approval or compliance.

This phenomenon of having all channels to have increment was mainly due to the unreliable baseline establishment. The baseline establishment was affected by the use of a muscle relaxant for intubation, which had not worn off fully by the time the MEP baseline is established. Some of the anaesthetists even use inhalational agents during intubation, and this will interfere with stable MEP baseline establishment. In Sunway Medical Centre, a one-level lumbar discectomy decompression procedure takes about 2 hours. The most ideal baseline should be established before decompression is done. But the problem is that, as shown in the example in Figures 1 and 2, the actual response was only obtained after the decompression is done, indicated by the global increments throughout all channels.

However, MEP can still be considered a prognostic tool by considering the following recommendations by the authors of this paper:

- Identify the problematic myotome based on presurgery clinical evaluation
- The TIVA protocol is the preferred anaesthesia throughout the surgery. If possible, the anaesthetist should intubate the patient without using inhalational gas
- Use higher stimulus intensity and number of trains if it is difficult to obtain observable MEP response, and lower down the stimulus intensity once the response amplitude is increasing when the surgery is progressing and the muscle relaxant effect is fading
- Request to stimulate MEP before decompression starts
- Observe the global behaviour of the MEP responses. Even if there are amplitude increment on the control channels (channels which are not the problematic myotome), the increment on the symptomatic myotome should be in higher percentage compared to that on the control channels. This may indicate improvement to the functional outcome of the patient
- Point (e) above should consider that all of the factors that could affect the MEP response as presented in Section 2.1 are not the cause of the assumption on improvement

Once we know the symptomatic myotome as stated in point (a) above and monitor it through MEP, we can observe visually the difference between the final reading and the initial baseline reading. If the initial and the final response makes prediction difficult as shown in Figures 1 and 2 as the responses heightened globally, we can still visually compare the symptomatic myotome against the other controlled channels. This means that the symptomatic myotome's improvement should be more significant compared to that of the other asymptomatic channels hence suggesting actual functional improvement.

The article "Transcranial Electrical Motor Evoked Potential in Predicting Positive Functional Outcome of Patients after Decompressive Spine Surgery: Review on Challenges and Recommendations towards Objective Interpretation" was retracted in 2023. Reasons: signs of a paper mill; suspected computer-generated content; unreliable results or conclusions; lack of ethics approval or compliance.

Point (b) is almost true for all of the surgeries that require IONM in Malaysia because of the increasing awareness among the anaesthetists of the need of TIVA for stable monitoring. However, the anaesthetists still have their own techniques used during intubation. Some of the anaesthetists are comfortable of using inhalational agents during intubation and will only switch to TIVA once the patient is positioned and draped. This will prolong the establishment of a reliable MEP baseline. A monitoring technician can only advice, but the anaesthetists will make their own decisions on what suits them and the patients best.

Point (c) is proposed because the adjustment of stimulus parameters as mentioned in Section 2.1.2 could help to establish a proper baseline if the MEP is affected by the muscle relaxant and inhalational agents used during intubation. Point (d) emphasizes on the important of communication between the IONM technician and the surgeon. If the surgeon is honest in utilizing the feedback from the IONM technology, the IONM technician should be allowed to request to do their tests (MEP more importantly because MEP stimulation causes the patient's body movement) at the times that suit their needs. Sometimes, requesting to test MEP just before the decompression starts will help to prolong the time needed for the anaesthesia from intubation to wear off, hence producing a stable MEP baseline. This will help the comparison between before and after decompression more reliable.

We propose that point (e) in the recommendations above should be assisted with signal processing and algorithm that could identify the global MEP response pattern of a patient during surgery, allowing the identification of significant improvement pattern on the problematic myotome. This can be done if more MEP parameters can be extracted and calculated compared to just relying on peak-to-peak amplitude or AUC as presented in studies mentioned in Section 2.

## 4. Conclusions

In this study, improvement to the MEP responses after surgical manipulation to the affected surgical sites from various levels of the spinal cord is shown in Section 2 to be highly corresponded to the positive functional outcome of the patients. This indicates that improvement to the MEP responses intraoperatively is reliable to be used as a prognostic tool and a valuable indicator to the surgeons during the surgery.

The article "Transcranial Electrical Motor Evoked Potential in Predicting Positive Functional Outcome of Patients after Decompressive Spine Surgery: Review on Challenges and Recommendations towards Objective Interpretation" was retracted in 2023. Reasons: signs of a paper mill; suspected computer-generated content; unreliable results or conclusions; lack of ethics approval or compliance.

However, there was no specific indicator for improvement that could be used to replicate the same result as the authors in Table 1 did in their studies. We highlighted in Discussion an example problem that prolonged anaesthetic muscle relaxant fading causes unknown suppression to the MEP baseline, causing wrong justification of improvement postdecompression. In order to make use MEP indications as a prognostic tool, we propose that the factors affecting MEP as presented in Section 2.1 should be maintained without huge variability throughout the surgery in the best way possible.

As we presented in Section 3, these improvement criteria need to distinguish between the global MEP behaviour and the symptomatic myotome MEP behaviour. We reviewed in Section 2.1 various factors that could affect MEP parameters such as the polyphase of the signal, latency of the response's starting point, and the duration or the length of the response. Some of these parameters are also presented in the reviews as the alarm criteria. These parameters can be further studied to be used as improvement criteria. A machine learning algorithm can also be used to make use of the combination of the MEP parameters as a pattern that signifies improvement rather than just relying on a single parameter.

Although significant work has been made in addressing such issue, there is much more room for the development of MEP improvement and its prognostic value correlation by taking into account the MEP signal's parameters and the justification of choosing the improvement criteria in the future.

## Figures and Tables

**Figure 1:** Baseline MEP response of a patient from microendoscopic discectomy of the L4/L5 procedure. LM2 and RM2: bilateral vastus lateralis. LM3 and RM3: bilateral tibialis anterior. LM4 and RM4: bilateral abductor hallucis. LM5 and RM5: bilateral medial gastrocnemius.

**Figure 2:** MEP response of a patient from microendoscopic discectomy of the L4/L5 procedure after decompression is performed. LM2 and RM2: bilateral vastus lateralis. LM3 and RM3: bilateral tibialis anterior. LM4 and RM4: bilateral abductor hallucis. LM5 and RM5: bilateral medial gastrocnemius.

**Table 1:** Summary for the reviews of the significance and the prognostic values of the MEP response improvement intraoperatively.

No.	Reference	No. of samples	IONM modalities used	Stimulation parameters	Muscles used to monitor MEP	Improvement criteria	Results
1	Barley et al. (2010)	One (15 months old boy)	TcMEP and SSEP	C1.-C2 scalp electrode positioning, current stimulation (145 mA to 187 mA for the left extremities and 175 mA to 200 mA for the right extremities)	Bilateral quadriceps femoris, tibialis anterior, gastrocnemius, sphincter, abductor pollicis brevis, abductor hallucis	Not mentioned	TcMEP response of the left APB had increment in amplitude. The patient had observable left upper extremity improvement

2	Voulgaris et al. (2010)	25 (2 had no IONM results)	TcMEP, EMG	C1–C2 with multipulse current stimulation, 0 mA to 200 mA, stimulus duration 0.2 ms to 0.5 ms	Not mentioned	>50% MEP amplitude improvement	17 patients with >50% improvement had better VAS score improvement

3	Rodrigues et al. (2011)	One (case report)	SSEP, MEP, and free-running EMG	C3-C4 stimulation	Not mentioned muscles' names specifically but monitoring covered L3-S2 myotomes	Not mentioned	MEP improved as much as 30%, and patient had returned to sports

4	Raynor et al. (2013)	386 patients had IOM signal improvement out of 12375 patients that had spinal surgeries over 25 years	DNEP, TcMEP, spontaneous EMG, triggered EMG, dermatomal SSEP	C3-C4 TcMEP scalp electrode stimulation montage	Upper extremity TcMEP was recorded from the deltoid, flexor/extensor carpi radialis, and/or abductor digiti minimi/abductor pollicis brevis. Lower extremity TcMEP was recorded from the anterior tibialis, medial gastrocnemius, and/or extensor hallucis longus	Not mentioned	The results did not mention specifically TcMEP improvement, but out of the modalities used, 88.7% patients had IOM signal improvement but one patient out of this percentage had permanent neurological deficit

5	Visser et al. (2014)	74 patients	TcMEP	Cz–Fz with monophasic stimulation and C3–C4 with biphasic stimulation	For the lower limbs: the quadriceps muscle (L2-L4), the tibialis anterior muscle (L4-L5), the hamstrings (L5-S1), or the gastrocnemius muscle (S1-S2). For cervical: the bilateral trapezoid muscle (C2-C4), the biceps (C5-C6), and the triceps muscle (C7-C8) of the arm; the extensor muscles of the forearm (C6-C7); or the abductor digitus V muscle (C6-C8)	>200% of amplitude increment	There is a correlation between the duration of symptom onset and the MEP improvement. MEP improvement can be accurate if the symptom onset duration is less than half a year

6	Wang et al. (2016)	59 patients that had cervical myelopathy underwent laminoplasty or laminectomy	MEP and SSEP	Not mentioned	Not mentioned	Not mentioned	Patients that had MEP signal improvement had a significant mJOA improvement rate. MEP amplitude was found to be a more accurate parameter compared to MEP latency in predicting surgery outcome

7	Dhall et al. (2017)	32	EMG, MEP, SSEP (not used for the study)	100 V–1000 V constant voltage stimulation, C1–C2 anodal stimulation, double train with a total of 9 pulses, 50 ms pulse width, 1.7 ms interstimulus, 13.1 ms ISI	Not mentioned	Comparison with the AIS grade and BASIC score of MRI images	MEP outcome (present) highly correlated with the better AIS grade and BASIC grade

8	Piasecki et al. (2018)	18	MEP, SSEP (not used for the study)	50 V–150 V C1–C2 biphasic stimulation, 5 to 7 train pulses, 500 Hz, 1 ms interstimulus pulse	1 upper limb muscle (control), bilateral tibialis anterior/bilateral abductor hallucis	>20% of AUC MEP, >50% of ZCQ score	The MEP improvement was related to the early follow-up functional outcome

9	Wi et al. (2019)	29 patients had improvement of IONM signals out of 317 cases	MEP and SSEP	Not mentioned	Upper extremity TcMEP was recorded from the deltoid, triceps, and thenar muscles. Lower extremity TcMEP was recorded from the anterior tibialis and abductor halluces	Comparison with MISS, SF-36, JOA, NDI, and Oswestry Disability Index	The patients with MEP improvement had a better MISS improvement rate while the patients with SSEP improvement only had a better SF-36 improvement rate

10	He et al. (2020)	One (case report)	MEP and free-running EMG	Not mentioned	Bilateral iliopsoas, rectus femoris, tibialis anterior, and medial gastrocnemius	Not mentioned	MEP improvement aligned with the patient's relieved symptoms

The article "Transcranial Electrical Motor Evoked Potential in Predicting Positive Functional Outcome of Patients after Decompressive Spine Surgery: Review on Challenges and Recommendations towards Objective Interpretation" was retracted in 2023. Reasons: signs of a paper mill; suspected computer-generated content; unreliable results or conclusions; lack of ethics approval or compliance.

## Data Availability

All the data are available from the list of references. Data presented in Figures 1 and 2 were collected from Sunway Medical Centre, Malaysia, upon medical ethics approval.
